# Application of Neural Network Algorithm in Medical Artificial Intelligence Product Development

**DOI:** 10.1155/2022/5413202

**Published:** 2022-06-08

**Authors:** Yineng Xiao

**Affiliations:** School of Health Humanities, Peking University, Haidian District, Beijing, China 100191

## Abstract

With the continuous deepening of artificial intelligence (AI) in the medical field, the social risks brought by the development and application of medical AI products have become increasingly prominent, bringing hidden worries to the protection of civil rights, social stability, and healthy development. There are many new problems that need to be solved in our country's existing risk regulation theories when dealing with such risks. By introducing the theory of risk administrative law, it analyzes the social risks of medical AI, organically combines the principle of risk prevention with benefit measurement, and systematically and flexibly reconstructs the theoretical system of medical AI social risk assessment. This paper has completed the following work: (1) reviewed and sorted out the works and papers related to medical AI ethics, medical AI risk, etc., and sorted out the current situation of medical AI social risk regulation at home and abroad to provide help for follow-up research. (2) The related technologies of artificial neural network (ANN) are introduced, and the risk assessment index system of medical AI is constructed. (3) With the self-designed dataset, the trained neural network model is utilized to assess risk. The experimental results reveal that the created BPNN model's error is relatively tiny, indicating that the algorithm model developed in this research is worth popularizing and applying.

## 1. Introduction

Under the rapid development of science and technology, AI has been applied in various fields. Medicine, as a field closely related to human beings, has naturally also been impacted. While countries in the world are constantly refreshing their understanding of AI, they are also constantly changing seize the opportunity in this new field [1, 2]. Since the outbreak of the “new crown” epidemic in 2020, more and more people's values have been greatly changed, and more attention has been devoted to the medical field. With the gradual penetration of AI, its intersection with medical undertakings will definitely become the focus of society, and this intersection has also emerged. AI has shown broad application prospects in medical diagnosis, data statistics, health monitoring, etc., which greatly improves the efficiency of diagnosis and treatment activities and brings a lot of convenience to human beings, but related problems are also accompanied [3, 4]. Western countries have begun to take measures to solve this problem, such as the “Robot Civil Law Rules” passed by the European Parliament and the “Restatement of Tort Law” passed by the United States, etc., which specifically introduced various measures to deal with AI. As a country that makes laws, due to the lag in legislation, the current legal system has not been perfected for new problems that may arise from AI, and the academic community also lacks a unified theoretical system. If the legal system in this area is not improved in time, it will inevitably hinder the advancement of artificial intelligence in the medical field [5]. Medical institutions, medical professionals, patients, designers and producers of medical AI, and other parties are all involved in the study, development, and implementation of medical AI products, making the ethical challenges raised by AI's use in medicine extremely complex. If we wish to improve human health, we must think about and act on the ethical challenges highlighted by medical AI. The ethical implications of medical technology can be viewed in two ways. The source of ethical worth is people. The ethical link between science and technology, people, and society is also what we research. The advancement of science and technology and the spirit of humanism must thus be integrated. It is certain that the negative impacts of science and technology will arise if the progress of science and technology is not guided by literary values. As a result, the reasonable use of artificial intelligence in the medical area needs ethical guidelines. Ethical risk governance mechanisms for medical AI should be promoted in the second step. Ethical questions are typically raised late in the game, resulting in a paucity of future ethical study [6]. This study, conducted in the contemporary age, examines the issues and causes associated with the use of medical AI and makes some recommendations and solutions in an effort to address some of the ethical concerns raised by this technology. The Civil Code stipulates that medical personnel shall bear tort liability, and medical institutions shall bear vicarious liability in violation of industry regulations or legal norms. Producers and sellers bear product liability due to product defects, but it is difficult to have a unified conclusion on how to position AI. The reason why there are many disputes is that my country's current legal system is blank in this regard. This article will draw on the legislative experience of foreign AI in the medical field to put forward risk assessment suggestions for the development of medical AI products in my country.

Facing the focus of domestic controversy, this article will combine various viewpoints in the academic circles and classify them according to the degree of intelligence of artificial intelligence. Use the intelligent level to locate its position in the medical field to explore new legal regulation paths and provide important opinions on various issues of artificial intelligence medical care [7]. AI has a broad space for development in real-time health monitoring, diagnosis and treatment data statistics, drug development experiments, etc., and can even respond faster than medical staff. However, AI has the characteristics of unpredictability and complexity, coupled with its strong learning ability and replication ability, which makes it have a certain degree of autonomy. This also exacerbates the uncertainty of future accidents [8, 9]. At the same time, intelligent programs inevitably have technical loopholes in the design process, which will also increase the probability of security risks and cause social conflicts. Therefore, the practical significance of this paper is to use the neural network algorithm to conduct reasonable risk assessment in the development of medical AI products, in order to reduce the occurrence of medical AI infringement cases.

The paper structures are as follows: Section 2 discusses the related work.  Section 3 defines the various methods of the proposed work.  Section 4 analyzes the experiment and analysis.  Section 5 concludes the article.

## 2. Related Work

Regarding the definition of artificial intelligence in the medical field, scholars have little controversy. Theoreticians generally believe that artificial intelligence is the intention of human beings to create intelligent machines that are close to humans, so that intelligent machines can replace medical personnel to complete various diagnosis and treatment activities, including health care, real-time monitoring, diagnosis and treatment data statistics, drug development trials, and intelligent surgical diagnosis. It is essentially a branch of computer science, and this science is then used in the medical field to provide medical services that are equivalent to or even greater than the responsibilities of medical personnel [10]. Reference [11], under the influence of foreign examples of “surgical robots,” concretized AI as intelligent medical robots and provided medical services based on AI technical means. The “intelligent technology + medical service” model has become a reality, which also enables precision medicine to provide solutions to the medical problems of an aging society in the future while reducing operating costs. From the perspective of AI medical infringement and the legal and ethical issues involved, scholars divide AI social risks into three categories: ethics, polarization, and regulation [12]. Ethical risk mainly refers to the passive or active breaking of human ethical relationship in the process of AI development, so that people have to reexamine and plan the ethical relationship. Since developers develop AI based on their own ethical concepts, AI inevitably has the basic value orientation of human beings, so how to control the adverse effects of developers in advance in the research and development stage has become the focus of AI regulation. With the development of AI to superintelligence, AI has replaced humans in many fields such as simple repetitive work, high-risk work, and companion services. It has changed from the object of human behavior to the same subject as human beings. Whether artificial intelligence can obtain legal subject qualification has become the main point to regulate its social risks [13]. Polarization risk mainly refers to the high development of artificial intelligence, although it can solve the existing problems of resource shortage and uneven distribution and liberate part of the simple and repetitive or high-risk labor force. However, the data and information that provide the basis for artificial intelligence are controlled by a small number of people, which will lead to the possibility of polarization of resources and wealth. The big data that artificial intelligence relies on is the result of detailed monitoring and analysis of personal information, so that individuals are completely exposed to the computer. Once there is a problem with the storage and confidential components of the computer, personal information will be in a difficult situation to protect [14]. Regulatory risk mainly refers to the phenomenon of excessive attention to economic benefits and neglect of civil rights that may occur in the process of national regulation of AI. In the process of economic development, developers who formulate AI software standards and write codes have absolute control over AI. Due to the confidentiality of AI programming by developers, coupled with the inducement of excessive pursuit of commercial interests, and the deviation of their own ethical values, the country will involuntarily tilt towards the research and development side in the process of AI regulation, resulting in citizens unable to effectively maintain legitimate interests. For AI social risk regulation, scholars generally agree to regulate it on the basis of the principles of justice, fairness, science, and rationality [15]. Ethical and moral regulation and legal regulation have become two important means of AI social risk regulation.

Ethics and ethics regulation requires that the ethical and ethical norms that it needs to follow be incorporated into the programming at the beginning of AI research and development and solve problems from the source. Legal regulation necessitates that the entire process of AI research, development, and application, as well as all relevant individuals involved, be restrained on the basis of solid legislation and effective law enforcement, which is an effective measure to avoid social problems created by AI [16]. In general, foreign AI development strategies mainly include consolidating the theoretical foundation of AI, building an AI security system, accelerating supporting legislation, and promoting international cooperation in AI research and risk regulation [17]. The British National Medical Service System has the world's leading medical level and is the leader in the development of medical AI in the United Kingdom. Its medical AI development experience is of great significance to my country [18]. The mid- and long-term health service system development plan released by it outlines the future development direction of UK medical AI from six aspects: service model innovation, reducing health inequality, promoting quality of care, providing employee support, realizing digital transformation, and improving investment utilization efficiency, including medical AI empowerment and empowerment, promoting medical AI clinical diagnosis and treatment application, and using medical AI to improve the safety and efficiency of population health management [19]. The US government has a relatively deep understanding and cognition of the current situation and development prospects of AI. “Preparing the Report for the Future of AI” analyzes and predicts the development of AI in the country and the world, points out the future research direction of AI and its possible social risks, and puts forward constructive countermeasures with suggestions. At the same time, the U.S. Congress has also actively paved the way for the development of AI and has promulgated many AI-related bills, which reflects the high attention of the American legal community to the development of AI. Although these policies and bills do not directly involve medical AI, they delineate a framework for the development of AI, which indirectly guides the development of medical AI and lays a foundation for regulating the social risks it brings [20–23].

## 3. Method

In the “Method” section, we define the basic theory of artificial neural network, risk assessment system for medical AI product development, data normalization, and parameter settings of the model in detail.

### 3.1. Basic Theory of Artificial Neural Network

#### 3.1.1. Artificial Neural Network Principle

ANN, an information processing system that replicates the structure and operation of a human brain, was built using modern neurobiological research. It also has the mental faculties of thinking, absorbing new information, and remembering what it has learned. A process of information processing can be viewed as a nonlinear mapping from the input space to the output space. Nonnormal distribution and nonlinear risk assessment issues may be solved efficiently by altering weights and thresholds to “learn” or discover the connection between variables. While each neuron in an ANN may be thought of as a fundamental operating unit, the method in which it processes information is not linear, and this is why ANNs are so complicated. The contact between these neurons also facilitates the processing of information across the whole neural network. The artificial neuron model is shown in Figure 1.

The *j*^th^ neuron in Figure 1 imitates the three most basic and important functions of biological neurons: weighting, summation, and transfer, where *x*_1_, *x*_2_, ⋯*x*_*n*_ represent the input from the neuron, *w*_*j*1_, *w*_*j*2_, ⋯*w*_*jn*_ represent the connection strength between the neuron and the *j*^th^ neuron, that is, the weight. *μ* is the threshold, which mainly adjusts the input and output of neurons. *f* is the transfer function. *y*_*j*_ is the output of the *j*^th^ neuron. Among them, the net input value *s*_*j*_ of the *j*^th^neuron is:

(1) $$\begin{array}{c} s_{j}=\overset{n}{\underset{i=1}{\sum }}w_{ij}*x_{i}+\mu =W_{j}X+\mu . \end{array}$$

After the net input *s*_*j*_ passes through the transfer function *f*, the output of the *j*^th^ neuron is obtained:

(2) $$\begin{array}{c} y_{j}=f\left(s_{j}\right)=f\left(\overset{n}{\underset{i=1}{\sum }}w_{ij}*x_{i}+\mu \right)=F\left(W_{j}X\right). \end{array}$$

Just as biological cells have the limit of information carrying, the signals transmitted by artificial neurons cannot increase indefinitely, and there must be a maximum value, where *f* should be a monotonically increasing bounded function.

ANN's learning and working phases are divided into two stages. To train a neural network, input and output data are fed into the network throughout this phase of development. Make the most of your network's settings. The network is given a new set of input samples as variables, and the learnt rules for processing yield new output results. In the working stage, a trained neural network looks like this. Self-learning and self-adaptation are other characteristics of the ANN, which may modify the weight values of neurons at each level as it learns to better suit the needs and requirements of its environment. In most cases, the neural network may be trained using two alternative ways. There are two types of algorithms: one utilizes a sample standard to modify the weight coefficients of each neuron to accomplish the goal of categorizing or mimicking the sample data; the other uses a neural network to learn. An algorithm with no tutor is another option, which merely describes how to learn. Depending on the input signal, the substance of the lesson changes. Environmental features and laws are discovered and stored by the system. The connection weights are also automatically adjusted. In order to group and aggregate input samples, this learning method is closer to the function of the human brain.

#### 3.1.2. Characteristics of Artificial Neural Network

Human brain neural networks may be modelled, simplified, and abstracted, and then used as a starting point for an ANN, which is built on this fundamental knowledge. In a similar way to the human brain, it can self-adapt, self-organize, and self-learn. It possesses strong intelligence qualities and has been effective in addressing numerous tough issues in the fields of pattern recognition, combinatorial optimization, and prediction. In general, ANN has the following characteristics:

1. It is quite good at nonlinear mapping

For a neural network to operate, it must be able to map data from the input layer to the output layer. Theoretically, any complicated nonlinear mapping may be realized by an ANN with three or more layers and sufficient hidden layer neurons, making it especially ideal for handling issues involving complex internal mechanics.

(2) Strong mathematical skills

Strong mathematical skills, as well as the capacity to solve real-world situations, distributed parallel processing, associative memory extraction technique, and complete activation of relevant neurons are used to extract information from external stimuli and input data in this system. The rules of the learning samples are adaptively taught, and the memory rules are stored using the “tutored” learning approach. The model can employ the prestored rules from the partial information and noise interference when a fresh random sample is added. The sample information is associatively memorized to achieve complete original information recovery, with good fault tolerance and strong anti-interference ability. It is especially suitable for the recognition of complex patterns with complex content and inconspicuous features.

(3) Strong sample identification and classification ability

The powerful nonlinear processing capability enables the neural network to handle the data classification of nonlinear samples well. As a nonlinear optimization algorithm, neural network has powerful optimization computing power; it can find a set of parameter combinations under known constraints, so that the objective function can quickly reach the minimum value.

(4) Good generalization ability

The neural network adopts the learning algorithm of global approximation and has good generalization ability. The network is highly trained and can tackle similar challenges in real time.

#### 3.1.3. Artificial Neural Network Model

Various ANN models, such as the BPNN model, the RBF neural network model, and the self-organizing mapping neural network model, have been established in the development of neural networks. This approach uses error back propagation, which is a hierarchical neural network made of an input layer, one or more hidden layers, and a final output layer. Layers of neurons are linked to each other like human nerve cells, and each layer has a certain number of neurons in it. Each layer of neurons is devoid of any connections. First, the input signal is sent from the input layer to the hidden node, where it is processed by the transformation function before being sent to the output node, where it is supplied as the final output result of the system. The number of network layers and the number of nodes in each layer are shown to have a positive correlation with the network's fitting accuracy. Increased network layers may enhance fitting accuracy, but the network becomes more complex, and training time goes up. There is a three-layer neural network structure according to the Kolmogorov theory, which can approximate any continuous function or accurate data classification with the precision of the mean square error and handle most real-world issues under specific circumstances for *ε* > 0. Linear data processing is also the most prevalent challenge. The network structure of the three-layer back-propagation neural network (BPNN) is shown in Figure 2.

In this network structure, the input vector is *X* = (*x*_1_, *x*_2_, ⋯*x*_*n*_)^*T*^, and the output vector of the hidden layer is

(3) $$\begin{array}{c} O_{k}=f\left(\text{ne}{\text{t}}_{k}\right). \end{array}$$

*Y* = (*y*_1_, *y*_2_, ⋯*y*_*m*_)^*T*^, the output layer vector is *k* = 1, 2 ⋯ *l*, and the expected output vector is *D* = (*d*_1_, *d*_2_, ⋯*d*_*l*_)^*T*^.

(4) $$\begin{array}{c} \text{ne}{\text{t}}_{k}=\overset{m}{\underset{j=o}{\sum }}w_{jk}y_{j}. \end{array}$$

The weight matrix between the input layer and the hidden layer is represented by *V*, *V* = (*v*_*l*1_, *v*_*l*2_, ⋯*v*_*mn*_)^*T*^, where *v*_*mn*_ represents the weight vector of the *n*th neuron in the hidden layer corresponding to the *m*th input layer neuron. The weight matrix between the hidden layer and the output layer is represented by *W*, *W* = (*w*_*il*_, *w*_2*l*_, ⋯*w*_*lm*_)^*T*^, where *w*_*lm*_ represents the weight vector of the first output layer neuron corresponding to the *m*th hidden layer neuron. For the output layer:

(5) $$\begin{array}{c} O_{k}=f\left(\text{ne}{\text{t}}_{k}\right)\left(k=1,2,\cdots ,l\right);\text{ne}{\text{t}}_{k}=\overset{m}{\underset{j=o}{\sum }}w_{jk}y_{j}\left(k=1,2,\cdots ,l\right). \end{array}$$

For the hidden layer:

(6) $$\begin{array}{c} y_{j}=f\left(\text{ne}{\text{t}}_{j}\right)\left(j=1,2,\cdots ,m\right),\text{ne}{\text{t}}_{j}=\overset{n}{\underset{i=o}{\sum }}v_{ij}x_{i}\left(j=1,2,\cdots ,m\right). \end{array}$$

The transfer function *f*(*x*) of the hidden layer and the output layer is a unipolar or bipolar Sigmoid function with continuous derivable characteristics:

(7) $$\begin{array}{c} f\left(x\right)=\frac{1}{1+e^{-x}}. \end{array}$$

The algorithm learning steps of BPNN are as follows:

1. Select a part of the overall sample as a training sample, and input its information into the network
2. The sample information is output by the output layer after being processed by the hidden layer of the network
3. Calculate the error value between the actual output and the expected output of the network
4. Reverse calculation from the output layer to the first hidden layer, and adjust the weights of the entire network according to the principle of error reduction
5. Repeat the above steps until the total error of the network reaches the target error value. After the repeated training of the above steps, the connection weights between the nodes of the network are completely confirmed, that is, the BPNN is trained. At this time, it can be used to identify and predict unknown samples

### 3.2. Risk Assessment System for Medical AI Product Development

With the continuous development of medical artificial intelligence, the distortion of medical data collection and the leakage of medical data, the unemployment of simple labor force and the increased medical burden of patients, the influence of scientific diagnosis and treatment and the aggravation of unequal distribution of medical resources, and other social risks will pose a huge threat to the benign development of society. At this point, all governments are working hard to create medical AI, as well as finding efficient strategies to manage the social hazards that come with it. However, in theory, the administrative laws and regulations governing medical AI social hazards are not very mature, and there are a number of issues. In practise, the merger of old administrative law leads to numerous loopholes. This paper analyzes the problems faced by the medical AI social risk administrative law regulation and combines the administrative process theory and the risk administrative law theory to build a basic theoretical framework for the social risk administrative law regulation of medical AI product development. The fundamental cognitive orientation of AI social risk administrative law regulation, the regulatory process monitoring, and the fundamental principles must be followed. And based on this, it analyzes and responds to the problems faced in the practice of medical AI social risk administrative law regulation.

#### 3.2.1. Risk Assessment

Strengthening medical AI social risk regulation scientific and rational risk assessment is to use facts and assumptions to estimate the probability that a special management decision will cause harm to human society. When human beings face uncertain social risks, risk assessment provides decision-makers with an orderly and clear basis for social risk regulation through scientific monitoring and analysis methods, combined with the opinions of various stakeholders. Risk assessment is the scientific basis for administrative agencies to regulate medical AI social risks. The National Academy of Sciences of the United States has made a scientific division of risk assessment in the book “Federal Government Risk Assessment; Management of the Process”, which includes: hazard cognition, through scientific experiments to determine whether there is a real hazard in the assessment object; hazard degree confirmation, determination degree of damage to humans in subjects was assessed at different doses; exposure assessment, by calculating and simulating the hazard of exposing people to such risks by calculating the intensity and frequency of human exposure to dangerous substances; risk estimation, analyzing relevant information and making risk determinations. Risk assessment is mostly based on the conclusions reached through scientific study by professional and technical professionals. Problems have developed in risk assessment in terms of technology, standards, authority distribution, assessment candidates, and public disclosure in the social risk regulation of medical AI. The reason is that the science used as the assessment scale is unstable. The instability of science is first reflected in the uncertainty of science itself. Science is developing gradually, and it is difficult to draw conclusions about the science and technology of a certain period. Secondly, it is reflected in scientists. On the one hand, scientists are limited by scientific development, and on the other hand, because of their own risk perception differences and political and economic influences, it is difficult to draw definite, objective, and rational conclusions in the evaluation. The risk administration law provides ideas for solving the instability of science through research on science and public participation, that is, introducing risk communication in the process of risk assessment.

#### 3.2.2. Risk Communication

Strengthening medical AI social risk regulation rational public risk communication is not equal to simple information disclosure. It is a process of information sharing and opinion exchange between administrative agencies and the public around a social risk topic. Risk communication actually runs through the whole process of medical AI social risk regulation. In order to unblock risk communication channels and achieve effective risk communication, the following issues must be clarified. The first is to ensure the authority of the publisher of the communication information. The same information is released by different individuals to produce completely different effects. When the administrative organ publishes relevant information for the purpose of regulating social risks, it must not only consider the professionalism of the relevant information but also consider your own integrity. Once the relevant information released by the administrative agency is confirmed to be false, the public's trust in it will be reduced and the effect of subsequent risk communication will be affected. The second is to enrich risk considerations. Administrative agencies should get rid of their extreme reliance on professional knowledge and incorporate the most common fairness and justice factors of public concern into the scope of risk considerations. The third is to pay attention to communication skills and to share risk-related information to the public as easily as possible, so that the public can participate in discussions on the basis of understanding; grasp the start time of risk communication. Starting too early will bring unnecessary panic to the public, and starting too late will lead to the suspicion of concealment. The timely initiation of risk communication will help safeguard citizens' right to know and to participate; it will help to eliminate the public's distrust of administrative agencies and mutual suspicion of various stakeholders caused by the concealment of information; it helps to ensure the continuous advancement of democracy in the process of risk regulation.

#### 3.2.3. Risk Identification Standards

Strengthening medical AI social risk regulation technology rational risk identification standards are the technical support for administrative agencies to regulate medical AI social risks and are also an important basis for risk assessment, communication, and management. Risk identification standards are authoritative, uncertain, professional, time-sensitive, and balanced. Legality means that the risk identification standards are formulated by the relevant institutions stipulated by law, and the risk identification standards have a legal basis. Uncertainty means that the risk identification standards are formulated under the uncertainty of scientific instability and social risks. As discussed above, it is extremely difficult to formulate risk identification standards under such circumstances. Professionalism means that although risk identification standards are formulated under the dual uncertainty of scientific and social risks, professional and technical personnel are still required to formulate them from a professional perspective. Timeliness means that the established criteria for identifying a certain type of risk will lose its validity over time, which is caused by the constant changes in social risks. Trade-off means that in the process of formulating risk identification standards, the framers have to weigh their interests. Risk identification standards have a direct impact on people's perceptions of risk and play a key role in risk regulation decisions made by decision-makers. Therefore, when formulating standards, it is necessary to weigh the interests of all parties involved in regulatory risks, and consider factors such as political needs and economic development. In this process, the important role of risk communication to ensure the objective and rationality of risk identification standards has also emerged.

#### 3.2.4. Risk Management

Strengthening medical AI social risk regulation to ensure rational risk management is the destination of medical AI social risk regulation. The purpose of administrative agencies to carry out risk management is to control the social risks of medical AI within an acceptable range and to minimize public losses and maximize public interests. The object of risk management of administrative organs is all risks that may threaten human society, mainly for those social risks that are identified as causing significant harm to human survival and development through risk assessment. With the continuous progress of society, the risk management of administrative agencies is bound to change from a power style to a communication style, and the risk management concept will also change from general management to refined management. Risk management is no longer an effort for the interests of some people, but to safeguard the legitimate rights and interests of all people. The administrative organ is no longer the only topic that must manage risk, and the latest development direction is for all stakeholders to work together.

According to the above evaluation of risk rules for medical AI product development, this paper designs an evaluation system that can be used for neural network experiments, such as Table 1. According to the evaluation results obtained by the input evaluation indicators, the risk of medical AI product development is divided into three levels.

### 3.3. Data Normalization

Since the hidden layer of the BPNN adopts a nonlinear and dimensional excitation function, it has the characteristics of saturated nonlinearity. If the difference between the input value of each neuron and the threshold is too large, the output of the neuron will fall in the saturation region, so that the actual output of the network is either the maximum value of the activation function or the minimum value of the activation function. The derivative value of the output tends to zero, resulting in a small change in the weights, which not only slows the learning speed but also makes the network difficult to converge. Therefore, in practical applications, in order to improve the training speed and sensitivity of the network and effectively avoid the saturation region of the excitation function, the value of the input data is generally required to be in the interval [0, 1], and it is necessary to normalize the input data. Commonly used normalization methods include linear function transformation method, logarithmic function transformation method, and arctangent function transformation method. This paper adopts the linear function conversion method:

(8) $$\begin{array}{c} x_{i}=\frac{x_{c}-x_{\min}}{x_{\max}-x_{\min}}, \end{array}$$

where *x*_max_ and *x*_min_ are the maximum and minimum values of the sample data, respectively, *x*_*i*_ is the original sample data, and *x*_*c*_ is the transformed data. The normalized data not only prevents the input data from falling into the saturation region, but also maintains the original characteristics of the data.

### 3.4. Parameter Settings of the Model

When using the BPNN model for risk assessment and analysis of medical AI product development, we should first set the corresponding parameters of the neural network to ensure the effective operation of the assessment model. Then, using the risk assessment index value and the evaluation sample's target value, train the network to produce an output value that is close to the target value. After repeatedly adjusting the parameter settings of the network, the model meets the requirements of the operation, and the neural network obtains the sample “knowledge” and stores it in the network weights and thresholds. At this point, a suitable risk assessment model is obtained, which can be used in practical work. Specific steps are as follows:

1. Setting of network nodes

After selecting a neural network, first set the network parameters, including the number of network layers and the number of nodes in each layer. The three-layer BPNN can solve most of the nonlinear data processing problems in reality, and it is the most common application. In this paper, the BPNN including the input layer, single hidden layer, and output layer is selected as the prediction model. In the simulation experiment, the number of nodes in the input layer is determined by the number of sample indicators, so the number of nodes in the input layer of the BP model in this paper is 14. The number of output layer nodes is 1. For the number of hidden layer nodes, there is still a lack of good theory as a guide, and different numbers of hidden layer nodes will form different neural network models. We need to perform constant and repeated debugging to obtain suitable network parameters, thus forming an effective risk assessment network model. The empirical formula used in this paper is as follows:

(9) $$\begin{array}{c} H=\sqrt{i+j}+a, \end{array}$$

where *H* is the number of hidden layer nodes, *i* is the number of output layer nodes, *j* is the number of output layer nodes, and *a* is a constant in the range [1–10]. Subsequently, the number of hidden nodes corresponding to the minimum network error will be determined by trial and error, thereby forming an initial three-layer BPNN model.

(2) Maximum training times

Set the maximum training times to 3000 times, that is, when the network training times reach 3000, stop training.

(3) Error accuracy

According to the software requirements and the needs of the model, the error precision set in this paper is le^−5^. When the error of the two iteration results is less than this value, the system will end the iterative operation.

(4) Excitation function

The input data of the neural network has been normalized and is in the range of [0, 1]. The excitation function of the hidden layer and the output layer of this paper is the logarithmic sigmoid function, that is, the Logsig function.

(5) Learning functions

Set to gradient descent momentum learning function (Learngdm).

(6) Training function

The gradient descent back-propagation algorithm function that adaptively adjusts the learning rate and adds a momentum factor is a combined optimization algorithm of the gradient descent method and the adaptive adjustment learning rate method. It has the characteristics of fast convergence speed, good learning effect, and high calculation accuracy, which improve the learning speed of the neural network and increase the reliability of the algorithm. The training function in this paper selects the traingdx algorithm.

(7) The error performance function

The error performance function of network convergence adopts the minimum mean square error value, and the target value is set as 0.0001.

## 4. Experiment and Analysis

In this chapter, we define the selection of evaluation samples, neural network model parameter selection and training, and test of neural network model in detail.

### 4.1. Selection of Evaluation Samples

My country's medical AI social risk legislation is still in the works, and the assessment of medical AI social hazards has flaws in terms of technology, norms, authority distribution, evaluation candidates, and public awareness. The current level of risk assessment technology development in my nation is insufficient to facilitate the effective development of assessment activities when compared to the actual needs of medical AI societal risk assessment. The cost-benefit analysis guides the standard risk assessment method. Due to the instability of the cost-benefit analysis itself, it is difficult to apply the traditional risk assessment method to the process of medical AI social risk assessment. Medical AI social risk assessment standards are an important part of medical AI social risk assessment, and an important basis for proving whether medical AI has social risks and whether it can be widely used in the medical field. Therefore, this standard cannot be limited to a single field, but should cover all areas where medical AI may have social risks. The current medical technology evaluation standards obviously cannot meet this requirement. The social risk assessment of medical AI mainly relies on professionals in related fields and administrative staff to form an expert group for assessment. On the one hand, there are many administrative staff, which is easy to reduce the scientific nature of the assessment; because the majority of them are drawn from universities and scientific research institutions in related subjects, and specialists are constantly in contact with one another, ensuring the impartiality and scientificity of evaluation viewpoints is difficult. Administrative activities relating to the social risk assessment of medical AI are not included in the scope that can be reported to the public, making public oversight of the social risk of medical AI impossible. Therefore, there is no assessment data suitable for this paper. According to the evaluation index system constructed in chapter 3, this paper designs an experimental dataset that can be used for neural network evaluation, which contains 320 datasets, 280 training sets, and 40 test sets.

### 4.2. Neural Network Model Parameter Selection and Training

In this paper, 12 different hidden layer nodes are used to train the network to determine the optimal network structure. After several simulation tests, the results are shown in Table 2.

It can be seen from Table 2 that when the number of hidden layer nodes is 8, after 200 network iterations, the network performance is 0.0000602, which meets the set error limit of 0.0001, and the error of the neural network model is the smallest at this time. Stop the iterative operation, and the network training is completed. At this time, after repeated debugging, the final selected network learning rate is 0.05, and the momentum factor is 0.95. The training effect is shown in Figure 3.

Therefore, this paper uses 8 hidden layer nodes to train and test the network, and builds a 12-8-1 three-layer BPNN model. To verify the application value of the constructed and trained neural network model, we must simulate the neural network constructed above using the training samples and compare the model's output results to the expected output results to see whether the simulation is right. If the correct rate is high, it means that the application of the neural network model constructed in this paper in judging the risk of medical AI development is scientific and effective and can be used in practice. To simulate the trained neural network, usually call the input variables of the sim function network in the neural network toolbox for simulation testing. After many simulation trainings, the error accuracy reaches the target value of 0.0001, and the network performance is 0.0000071526. It can be seen from Figure 4 that the constructed neural network model has a high-precision prediction and judgment ability.

The obtained training sample simulation results are shown in Figure 5.

### 4.3. Test of Neural Network Model

The neural network and simulation test constructed above are all derived from the training sample data, showing a good discriminative effect. The generalization effect of the model, that is, the discriminative effect of the nontraining sample data, needs to be tested to judge the promotion and application value of the model. This study simulates the neural network established above using the selected 40 sets of test sample data as input, then compares the model's output results to the expected output results to assess the simulation's accurate probability. For the simulation test, 40 groups of test sample data were entered into the trained neural network model, and its risk was assessed; 10 groups of data were chosen, and the results are presented in Figure 6. It can be seen from the experimental results that the error of the output results is very small, which shows that the application of the neural network model constructed in this paper in judging the development risk of medical AI is scientific and effective and has good promotion and application value.

## 5. Conclusion

AI technology in my country's medical field is still in the weak AI stage, and its research and development and application are still in the early stage, but AI has great potential in accelerating medical scientific discovery and transforming medical care. The era of “strong AI” may be close at hand. The application of technology in medicine is linked to human health and survival. Medical AI is difficult to implement. It is critical to comprehend the potential dangers and consequences of this new technology. Medical AI should be better regulated, and AI should be applied in the most efficient way feasible to ensure that the patient's experience and needs are prioritized. As a result, this article employs neural networks to assess risk in the development of medical AI and completes the following tasks: (1) reviewed and sorted out relevant works and papers on medical AI ethics, medical AI risks, etc. The current situation of regulation is sorted out to provide help for follow-up research. (2) The related technologies of ANN are introduced, and the risk assessment index system of medical AI is constructed. (3) With the self-designed dataset, the trained neural network model is utilized to assess risk. The experimental results reveal that the created BPNN model's error is relatively tiny, indicating that the algorithm model developed in this research is worth popularizing and applying.

## Figures and Tables

**Figure 1:** Artificial neuron model.

**Figure 2:** BP neural network structure diagram.

**Figure 3:** BP neural network training error curve.

**Figure 4:** Variation curve of training simulation error of neural network.

**Figure 5:** Training sample simulation results.

**Figure 6:** Test sample simulation results.

**Table 1:** Medical AI product development risk assessment system.

Index	Label
Weakening of doctors' practical ability	R1
Weakening of the moral responsibility of doctors	R2
Patient privacy violated	R3
The humanity of the patient is challenged	R4
The rights of patients cannot be guaranteed	R5
Lack of doctor-patient trust	R6
Weakening of humanistic care	R7
Influencing the scientific nature of patient care research	R8
Exacerbating the unequal distribution of medical resources	R9
Simple labor unemployment risk	R10
Risk of increased medical burden on patients	R11
Medical data collection distortion	R12
Risk of medical data breach	R13
Generate ethical and moral hazard	R14

**Table 2:** Training results for different numbers of hidden layer nodes.

Number of hidden layer nodes	Mean squared error
5	0.0000977
6	0.0000869
7	0.0000619
8	0.0000602
9	0.0000788
10	0.0000872
11	0.0000948
12	0.0000982
13	0.0000965
14	0.0000990
15	0.0000974
25	0.0000893
35	0.0000989
45	0.0000948

## Data Availability

The datasets used during the current study are available from the corresponding author on reasonable request.
